# Multimedia Real-Time Transmission Protocol and Its Application in Video Transmission System

**DOI:** 10.1155/2022/8654756

**Published:** 2022-05-23

**Authors:** Xinkan Zhang, Fufeng Chu

**Affiliations:** ^1^Minnan Science and Technology University, Quanzhou, Fujian 362332, China; ^2^Xiamen University Tan Kah Kee College, Zhangzhou, Fujian 363105, China

## Abstract

The aim is to provide corresponding quality of service (QoS) guarantee for real-time video data transmission. To ensure the high quality and smooth playback of video sequence at the receiving end, the design of multimedia transmission is made. In view of the shortcomings of selective frame loss, this paper adopts the active frame loss algorithm, which discards the nonkey frames according to the probability. With the increase of the frame loss rate at the transmitter, the proportion of decoded frames increases rapidly and reaches the maximum when the frame loss rate is 0.1. It is proved that active frame loss can control the bit rate more accurately to make full use of bandwidth resources and avoid the waste of bandwidth resources.

## 1. Introduction

With the increasing demand for network video, how to make users obtain good viewing effect when viewing network video has become a hot research topic [1]. Because the network video playback is subject to the user's equipment and network transmission, it brings adverse effects such as low definition or not smooth enough to the user's browsing. How to develop an adaptive video player and transmit appropriate video to users according to users' equipment performance parameters and network performance is an important research content in the field of adaptive video transmission [2]. Among many adaptive control methods of video transmission, selective frame loss has very low time complexity and good real-time performance, which can be applied in most occasions. However, most of the existing frame loss algorithms adopt the hierarchical rate adjustment method, which is equivalent to a coarse-grained bandwidth matching method, which makes the code rate and decoding quality change step by step, and cannot achieve the accurate matching with the channel bandwidth. Finally, this paper combines the active frame loss strategy by reducing the segment length and improves the parallelism of data transmission by reducing the number of transmitted video frames and giving up part of the bandwidth for the transmission of additional overhead caused by the increase of the number of video frame segments, so as to improve the real-time requirements of delay sensitive data transmission and achieves good results.

## 2. Literature Review

As the problems of traditional streaming media transmission methods become more prominent, adaptive streaming has gradually become the mainstream technology of video transmission, as shown in Figure 1, but there are few adaptive algorithms designed with new standards. This leaves room for competition among scholars [3]. Neil et al. proposed a buffer-based fuzzy logic control bit rate adaptive algorithm, according to the change of the buffer. The video bit rate is controlled according to certain rules [4]. Qi and others described a typical rate adaptive control algorithm based on slow change of playback [5]. Mok and others start from the quality of experience (QoE), through the analysis of the factors that affect the QoE value; a video bit rate adaptive algorithm is proposed; and the value of QoE is made the best [6]. Kim and others used the monitoring mechanism in the algorithm, every cycle, to monitor the available bandwidth in the network, the size of client cache data, and the amount of frame loss, as a parameter to determine the switching code rate, and when the current available bandwidth is lower than the current video stream bit rate, the average frame loss rate is greater than 10%, or when the remaining buffer length is less than the set active buffer length *B*_*a*_, the client switches to a lower video bit rate [7]; Verkatraman et al. introduced the concept of sliding window in the algorithm, based on the average download time in the sliding window, as a parameter to measure the state of the network, used the logistic equation, modeled the network throughput and rate reduction factor, limited the amplitude of the bit rate jump, maintained the video buffer within the equalization interval, and reduced the number of code rate switching [8]. Meng and others pointed out bandwidth estimation and bit rate selection as they are the core of the client-side bit rate adaptive algorithm and used Q learning enhanced learning algorithm to train a decision-making *Q* matrix; according to the current network status and buffer saturation, the *Q* matrix is referred to determine an action that can obtain the maximum return value; the algorithm can achieve higher bit rate level, less bit rate switching time, and balance the amount of buffered data [9]. Hassan and others used historical download data to predict the network bandwidth in the next stage, using the standard deviation method; replaced the original SF algorithm for the calculation of volatility parameters [10]; made the bandwidth prediction result smoother and slow down the occurrence of the “burr” phenomenon, and combined with the buffer management strategy to make the basis for the code rate decision, avoiding the shortcomings of relying on a single parameter as the code rate selection. The algorithm has high stability, but when the state of the cache is in the balance zone, even if the available bandwidth resources of the network become larger, the algorithm pursues stability. It will not switch to a higher level of video bit rate. Altaf et al. implemented the video bit rate switching algorithm in the OpenFlow network, using the OpenFlow network to be able to pass through the network controller, and obtained real-time traffic information of all switch ports. The accuracy and usability of the algorithm are improved, and the interference of other additional data is avoided [11]. But Mongay Batalla and others found that because when data are transmitted over the network, the network bandwidth will fluctuate greatly and only make bit rate decisions based on the throughput of the network. There is a certain degree of one-sidedness. If the cache state is not considered in the decision, it is likely to cause a series of buffer overflow and frequent bit rate switching, which will affect the user's viewing experience [12]. Hooft et al., according to the shortcomings of the current existing algorithms, proposed an algorithm that prioritizes caching. When the network changes significantly, priority is given to the client's cache status, and then according to the available bandwidth of the network, it is judged whether or not to switch the code rate [13].

## 3. Methods

### 3.1. The Best Frame Loss Rate and Its Determination

In the case of insufficient bandwidth, the method of actively discarding nonkey frames can significantly improve the decoding quality of video [14]. At that time, for each B frame sent, the probability Pdrop calculated by the following formula is discarded:

(1) P=drop2BWC−BWABWC.

The purpose is to adjust the data sending rate to match the bandwidth. In order to determine the probability Pdrop here, whether it is the parameter that maximizes the ratio of decodable frames, we need to examine the relationship between different frame loss rates and the ratio of decodable frames. Here, through the method of simulation experiment, the relationship between the frame loss rate and the ratio of decodable frames is studied, and the network topology is simulated. The video recording file Verbose_StarWarsIV.dat is still used here to generate data traffic, and the required transmission bandwidth is 320 kb. Our fixed network bottleneck link, that is, the link bandwidth between R1 and R2, is 304 kb, that is, 95% is needed to simulate the situation of insufficient bandwidth. Here, the frame loss rate Pdrop is adjusted from 0 to 0.2, and the change of the decodable frame ratio is observed [15]. The experimental results are shown in Figure 2. As can be seen from the figure, when the frame loss rate is 0, because the available network bandwidth is insufficient, the network is in a congested state, a lot of packet loss makes the frame. In the process of transmission, the dependence is destroyed. Although the available bandwidth reaches 95% of the required bandwidth, the proportion of decodable frames is only a little over 77%, and random packet loss has a serious adverse effect on the decoding quality of the video. As the frame loss rate at the sender increases, the proportion of decoded frames increases rapidly, and it reaches the maximum value when the frame loss rate is 0.1 [16]. When the frame loss rate is 0.1, the amount of data that the sender actively loses is 5% of the total video data because we only discard noncritical B-frames and the B-frame data volume accounts for half of the total data volume. Therefore, only 95% of the data is sent to the network, and the network is in a bandwidth matching state at this time. In the process of controlling the frame loss rate from 0 to 0.1, it is the process of adjusting the data transmission rate of the sender to match the bandwidth. Although the network is still congested during this period, but as the degree of congestion decreases, the forced random packet loss on the network is reduced, as shown in Figure 3. The adverse impact of random packet loss on video decoding is alleviated, and the proportion of decodable frames increases rapidly. When the control frame loss rate continues to increase from 0.1, because the data transmission rate is lower than the transmission capacity of the network, the packet loss rate is reduced to 0; at this time, as the total amount of data sent by the sender decreases, the video data received by the receiving end is also reduced accordingly. Therefore, the proportion of frames that can be decoded decreases as the frame loss rate increases. At this time, the network is under light load.

To sum up, for a certain available bandwidth, when it is insufficient to meet the minimum demand of video transmission, the maximum decodeable frame ratio can be obtained by determining the optimal frame loss rate and implementing the active frame loss strategy under the optimal frame loss rate. Here, the best frame loss rate is to match the data transmission rate with the network bandwidth. This also verifies the correctness of the formula for calculating the frame loss rate in our above algorithm. Using only the UDP protocol, the network can only provide best-effort services. This was originally designed for data service transmission, for video data with strong real-time performance, large data volume, sensitive to random data loss, and high requirements for transmission delay and jitter. The quality of its service cannot be guaranteed. In order to improve the quality of video data transmitted through traditional networks, IETF (Internet Engineering Task Force) formulated RTP and RTCP protocols in 1996, which provides a real-time transmission standard for the network [17, 18]. Real-Time Transport Protocol (RTP) is only responsible for the transmission of real-time data, is a data transfer protocol, and used for the transmission of multimedia data streams on the Internet. Real-Time Transport Control Protocol RTCP is used in the process of data transmission and provides feedback on network status and service quality for data senders. The RTCP protocol defines several datagrams as shown in Figure 4 to achieve its functions: the sender reports (SR), the receiver reports (RR), and the source description package (SDES). The conversation person leaves the package BYE and specific application package APP. Among them, the sender reports and the receiver reports are used for RTP participants to exchange statistical information with each other [19, 20].

### 3.2. Measurement and Improvement of Continuous Frame Loss

The selective frame loss algorithm is a “deterministic” algorithm. The certainty here means that when the control parameters are determined, for a certain video sequence, whether a frame is discarded is certain, generally, there will be no continuous frame loss, unless the algorithm specifically arranges. This may cause continuous frame loss. Continuous frame loss will cause jumps and interruptions in video playback at the receiving end and affect the quality of video playback. Number the B frames at different positions in a GOP, the first one is 1, the second is 2, the third is 3,…, the eighth is 8. Use probability *p*(*x*_*i*_) to represent the active frame loss algorithm. The probability that the frame number *i* is discarded and then the conditional probability *p*(*x*_*i*_+1*|x*_*i*_) means that when the frame numbered *i* is discarded, the probability that the frame numbered *i* + 1 is discarded [21, 22]. Obviously, the conditional probability *p*(*x*_*i*_+1*|* *x*_*i*_) can describe the continuity of dropped frames, the greater the probability, the greater the possibility of continuous frame loss, and the worse the uniformity. For different *i*, the conditional probability *p*(*x*_*i*_+1 *|* *x*_*i*_) is not necessarily the same, take its statistical average here, in order to measure the continuity of frame loss in an algorithm:

(2) $$\begin{array}{c} H\left(X_{i+1}\;|\;x_{i}\right)=\frac{\Sigma p\left(x_{i}\right)p\left(x_{i+1}\;|\;x_{i}\right)}{\Sigma p\left(x_{i}\right)}. \end{array}$$

Call *H*(*X*_*i*+1_*|x*_*i*_) the average conditional probability, the larger the value, the greater the possibility of continuous frame loss, the worse the uniformity of dropped frames. We use the average conditional probability *H*(*X*_*i*+1_*|x*_*i*_), in order to examine the uniformity of three different frame dropping algorithms, let the average frame loss rate be *P*. For each *B* frame, regardless of its number, all follow the same probability *P* [23, 24]. The discard probability is shown in Table 1.

At this time, because the discarding probabilities of each frame are independent of each other, the conditional probability is shown in Table 2.

According to formula (2), *H*(*X*_*i*+1_*|x*_*i*_)=*p*_*a*_ is calculated.

Considering that the rate adjustment needs to consider TCP friendliness and stability, here are two methods to set the optimal frame loss rate: the detection method and the model method. After using the RTCP protocol to obtain the state information of the network, the detection method imitates the additive growth of TCP according to the congestion state of the network and adjusts the setting of the frame loss rate according to the multiplicative reduction behavior: the formula rule is to calculate the effective bandwidth of the network according to the TFRC congestion control algorithm and then directly calculate and set the optimal frame loss rate according to the formula. Since the congestion control algorithms on which the two methods are based are both TCP-friendly rate control algorithms, the frame loss rate adjustment method here is also TCP-friendly.

## 4. Results and Analysis

In the method, we use an equal-probability frame loss algorithm, regardless of the number of each B frame, and all are discarded according to the same probability *p*_*a*_ [25, 26]. Although in comparison with Section 3, this algorithm is better than the uniformity of the arithmetic series probability of frame loss. The uniformity of frame loss proportional series probability is also good. However, the probability of continuous frame loss, especially the average frame loss rate *P*_*a*_, is still relatively high especially when it is relatively large. In order to improve the uniformity of dropped frames, consider the distance between the current frame and the last actively discarded frame and determine the size of the discarding probability. The closer the distance, the smaller the probability of discarding. The greater the distance, the probability of discarding is also greater, which reduces the possibility of continuous frame loss. The discarding probability of the current frame at this time is only related to the distance from the last dropped frame. We can use a Markov chain to design an algorithm that meets the above requirements. *k* is used to represent the distance between the current frame and the last actively discarded frame *S*={1,2,3,…} is the state space of Markov chain, so the one-step transition probability is specified as

(3) $$\begin{array}{c} p_{k,k+1}=\frac{1}{h^{k}}, \end{array}$$

where *h* > 1. There is

(4) $$\begin{array}{c} p_{k,1}=1-\frac{1}{h^{k}}, \end{array}$$

where *k* is the distance between the current frame and the last discarded frame. The one-step transition probability matrix of this model is

(5) $$\begin{array}{c} p=\left[\begin{array}{cccccc} 1-\frac{1}{h} & \frac{1}{h} & 0 & 0 & 0 & 0\\ 1-\frac{1}{h^{2}} & 0 & \frac{1}{h^{2}} & \; & \; & \;\\ 1-\frac{1}{h^{3}} & 0 & 0 & \frac{1}{h^{3}} & \; & \;\\ 1-\frac{1}{h^{4}} & 0 & 0 & 0 & \frac{1}{h^{4}} & \;\\ 1-\frac{1}{h^{5}} & 0 & 0 & 0 & 0 & \frac{1}{h^{5}} \end{array}\right]. \end{array}$$

*h* is a parameter corresponding to the average frame loss rate Pa, which can control the average frame loss rate. Obviously, *p*_*k*.*k*+1_=1/*h*^*k*^ represents the rate at which the previous frame is not discarded when the distance between the previous frame and the last actively discarded frame is *kp*_*k*.1_=1 − 1/*h*^*k*^ means that when the distance between the current frame and the last actively discarded frame is *k*, the probability of being discarded is high. The greater the *k*, the greater the probability of the current frame being discarded; the smaller the *k*, the smaller the probability of being discarded. The frame loss uniformity of active frame loss algorithm is improved. Next, we study the relationship between the control parameter *h* and the average frame loss rate *p*_*a*_. According to the one-step transition probability matrix P,

(6) $$\begin{array}{c} f_{11}^{1}=1-\frac{1}{h},\\ f_{11}^{2}=\left(\frac{1}{h}\right)\left(1-\frac{1}{h^{2}}\right),\\ \begin{array}{c} \ldots \ldots \end{array}\\ f_{11}^{n}=\left(\frac{1}{h}\right)\left(\frac{1}{h^{2}}\right)\cdots \left(\frac{1}{h^{n-1}}\right)\left(1-\frac{1}{h^{n}}\right), \end{array}$$

where *f*_11_^*n*^ is starting from state 1, probability of returning to state 1 for the first time after *n* steps, that is, the probability of discarding a video frame at intervals of *n* steps. So, there is an average number of steps that return to state 1, that is, the average interval between dropped frames is

(7) $$\begin{array}{c} =\sum_{n=1}^{\infty }nf_{11}^{n}=\left(1-\frac{1}{h}\right)+2\frac{1}{h}\left(1-\frac{1}{h^{2}}\right)+\cdots +\lambda \\ =1+\frac{1}{h}+\left(\frac{1}{h^{2}}\right)\cdots +\cdots \\ =\sum_{n=0}^{\infty }\frac{1}{h^{n\left(n+1\right)/2}}. \end{array}$$

And, because the average frame loss interval and the average frame loss rate *p*_*a*_, there is the following relationship:

(8) $$\begin{array}{c} \lambda =\frac{1}{p_{a}}. \end{array}$$

So, the relationship between the control parameter *h* and *p*_*a*_ is

(9) $$\begin{array}{c} p_{a}=\frac{1}{\sum_{n=0}^{\infty }1/h^{n{\left(n+1\right)}^{2}}}. \end{array}$$

Therefore, *p*_*a*_ is determined, and *h* is also determined. The relationship between the two is shown in Figure 5.

Now, use the improved algorithm and the equal-probability jade frame algorithm and compare the uniformity of dropped frames. Just look at *H*(*X*_*i*+1_ *|* *X*_*i*_), the larger the value, the worse the uniformity of frame loss; for the equal-probability frame loss algorithm,

(10) $$\begin{array}{c} H\left(X_{i+1}\;|\;X_{i}\right)=P\left(X_{i}\right)=P_{a}. \end{array}$$

For the improved algorithm of this paragraph,

(11) $$\begin{array}{c} H\left(X_{i+1}\;|\;X_{i}\right)=1-\frac{1}{h}. \end{array}$$

The relationship between *h* and *p*_*a*_ is determined by formula (9). We draw the *H*(*X*_*i*+1_ *|* *X*_*i*_) of the two algorithms under different average frame loss rate *p*_*a*_, as shown in Figure 6:

As can be clearly seen from the figure, in the case of the same average frame loss rate, the *H*(*X*_*i*+1_ *|* *X*_*i*_) of the improved algorithm is much smaller, and it can make the frame loss more even.

## 5. Conclusion

This paper proposes an improved method to determine the optimal frame loss rate. When the frame loss rate is 0, although the available bandwidth reaches 95% of the required bandwidth, the proportion of decodeable frames is only a little more than 77%. Random packet loss has a serious adverse impact on the decoding quality of the video. With the increase of the frame loss rate at the transmitting end, the proportion of decodeable frames increases rapidly and reaches the maximum value when the frame loss rate is 0.1 [27-28]. When the frame loss rate is 0.1, the amount of data actively lost by the sender is 5% of the total video data. Because we only discard non critical B frames and the amount of B frame data accounts for half of the total data, only 95% of the data is sent to the network. At this time, the network is in the state of bandwidth matching. The process of controlling the frame loss rate from 0 to 0.1 is to adjust the data transmission rate of the transmitter to match the bandwidth. The active frame loss algorithm may have continuous frame loss. In order to solve this problem, the concept of average conditional probability is used to measure the frame loss uniformity of a frame loss algorithm, and its calculation method is explained by an example. In order to reduce the probability of continuous frame loss events, the equal probability frame loss algorithm is improved to improve the uniformity of the frame loss algorithm. This paper studies the relationship between the control parameters of the improved algorithm and the average frame loss rate, gives the method to determine the control parameters, and verifies its correctness through simulation experiments. Finally, we compared two groups of experiments and investigated the average frame loss interval and frame loss interval variance of the two algorithms under the same network conditions. The conclusion shows that the improved algorithm greatly improves the uniformity of frame loss.

## Figures and Tables

**Figure 1:** Network development flow chart.

**Figure 2:** Decodable frame ratio.

**Figure 3:** Packet loss rate.

**Figure 4:** Schematic diagram of RTCP work.

**Figure 5:** The relationship between *P*_*a*_ and (*h*).

**Figure 6:** *H*(*X*_*i*+1_*|X*_*i*_).

**Table 1:** Discard probability.

*P*(*X*_1_)	*P*(*X*_2_)	*P*(*X*_3_)	*P*(*X*_4_)	*P*(*X*_5_)	*P*(*X*_6_)	*P*(*X*_7_)	*P*(*X*_8_)
*P*_*a*_	*P*_*a*_	*P*_*a*_	*P*_*a*_	*P*_*a*_	*P*_*a*_	*P*_*a*_	*P*_*a*_

**Table 2:** Conditional probability.

*p*(*x*_2_ *|* *x*_1_)	*p*(*x*_3_ *|* *x*_2_)	*p*(*x*_4_ *|* *x*_3_)	*p*(*x*_5_ *|* *x*_4_)	*p*(*x*_6_ *|* *x*_5_)	*p*(*x*_7_ *|* *x*_6_)	*p*(*x*_8_ *|* *x*_7_)	*p*(*x*_1_ *|* *x*_8_)
*P*_*a*_	*P*_*a*_	*P*_*a*_	*P*_*a*_	*P*_*a*_	*P*_*a*_	*P*_*a*_	*P*_*a*_

## Data Availability

The data used to support the findings of this study are available from the corresponding author upon request.

## References

[1] Siagian P., Fernando E. (2021). The design and implementation of a dashboard web-based video surveillance in openstack swift. *Procedia Computer Science*.

[2] Xu J., Dai J., Rao R., Xie H., Lu Y. (2016). Critical systems thinking on the inefficiency in post-earthquake relief: a practice in longmen Shan fault area. *Systemic Practice and Action Research*.

[3] Jia K., Li H., Yuan Y. (2017). Application of data mining in mobile health system based on apriori algorithm. *Journal of Beijing University of Technology*.

[4] Heffernan N. T., Ostrow-Korinn K. S., Kelly K. (2016). The future of adaptive learning: does the crowd hold the key?. *International Journal of Artificial Intelligence in Education*.

[5] Qi X., Zhao G., Shen L., Li Q., Pietikäinen M. (2016). Load: local orientation adaptive descriptor for texture and material classification. *Neurocomputing*.

[6] Mok R. K. P., Li W., Chang R. K. C. (2016). Irate: initial video bitrate selection system for http streaming. *IEEE Journal on Selected Areas in Communications*.

[7] Kim M., Kim H., Chung K. (2018). Video quality control scheme for efficient bandwidth utilization of http adaptive streaming in a multiple-clients environment. *Journal of KIISE*.

[8] Verkatraman S., Nam J. Y., Rao K. R. (1995). Image coding based on classified lapped orthogonal transform-vector quantization. *IEEE Transactions on Circuits and Systems for Video Technology*.

[9] Meng S., Sun J., Duan Y., Guo Z. (2016). Adaptive video streaming with optimized bitstream extraction and pid-based quality control. *IEEE Transactions on Multimedia*.

[10] Hassan M. M., Farooq U. (2016). Adaptive and ubiquitous video streaming over wireless mesh networks. *Journal of King Saud University - Computer and Information Sciences*.

[11] Altaf M., Khan F. A., Qadri N., Ghanbari M., Dudley S. E. (2017). Adaptive robust video broadcast via satellite. *Multimedia Tools and Applications*.

[12] Mongay Batalla J. (2016). Advanced multimedia service provisioning based on efficient interoperability of adaptive streaming protocol and high efficient video coding. *Journal of Real-Time Image Processing*.

[13] van der Hooft J., Petrangeli S., Wauters T., Huysegems R., Alface P. R., Bostoen T. (2016). Http/2-based adaptive streaming of hevc video over 4g/lte networks. *IEEE Communications Letters*.

[14] Hanca J., Braeckman G., Munteanu A., Philips W. (2016). Lightweight real-time error-resilient encoding of visual sensor data. *Journal of Real-Time Image Processing*.

[15] Kwon D., Kim J., Mohaisen D. A., Lee W. (2020). Self-adaptive power control with deep reinforcement learning for millimeter-wave internet-of-vehicles video caching. *Journal of Communications and Networks*.

[16] Zhang X., Toni L., Frossard P., Zhao Y., Lin C. (2019). Adaptive streaming in interactive multiview video systems. *IEEE Transactions on Circuits and Systems for Video Technology*.

[17] van der Hooft J., Petrangeli S., Wauters T., Huysegems R., Bostoen T., De Turck F. (2018). An http/2 push-based approach for low-latency live streaming with super-short segments. *Journal of Network and Systems Management*.

[18] Rodríguez A. C., Roda C., Montero F., González P., Navarro E. (2016). An interactive fuzzy inference system for teletherapy of older people. *Cognitive Computation*.

[19] Carlsson N., Eager D., Krishnamoorthi V., Polishchuk T. (2017). Optimized adaptive streaming of multi-video stream bundles. *IEEE Transactions on Multimedia*.

[20] Chae S.-H., Moon H.-M., Chung Y., Shin J., Pan S. B. (2016). Automatic lung segmentation for large-scale medical image management. *Multimedia Tools and Applications*.

[21] Şeref O., Razzaghi T., Xanthopoulos P. (2017). Weighted relaxed support vector machines. *Annals of Operations Research*.

[22] Almadani B. (2016). Qos-aware real-time pub/sub middleware for drilling data management in petroleum industry. *Journal of Ambient Intelligence and Humanized Computing*.

[23] Kim Y., Kim H., Chung K. (2018). Video quality maintenance scheme for improve qoe of http adaptive streaming service. *Journal of KIISE*.

[24] Huang S., Izquierdo E., Hao P. (2017). Adaptive packet scheduling for scalable video streaming with network coding. *Journal of Visual Communication and Image Representation*.

[25] Taha M., Canovas A., Lloret J., Ali A. (2021). A qoe adaptive management system for high definition video streaming over wireless networks. *Telecommunication Systems*.

[26] Frederick D. D. S., Junaid M. K. A., Jaison B., Rose A. J. T. (2018). Dynamic association and participant based adaptive streaming in small base station for live video conference on 5g networks. *Transactions on Emerging Telecommunications Technologies*.

[27] Kim M., Chung K. (2017). A video quality adaptation algorithm to improve qoe for http adaptive streaming service. *Journal of Kiise*.

[28] Mongay Batalla J., Krawiec P., Beben A., Wisniewski P., Chydzinski A. (2016). Adaptive video streaming: rate and buffer on the track of minimum rebuffering. *IEEE Journal on Selected Areas in Communications*.

